The article "Artificial Neural Network Model for Indoor Decoration Intelligence Calculation and Automation Design" was published in 2022. Journal: Comput Intell Neurosci.

# Artificial Neural Network Model for Indoor Decoration Intelligence Calculation and Automation Design

**DOI:** 10.1155/2022/2246211

**Published:** 2022-06-24

**Authors:** Yan Li

**Affiliations:** College of Art and Design, School of Anyang Institute of Technology, Anyang 45500, Henan, China

## Abstract

With the continuous development of science and technology, the indoor decoration industry has gradually changed toward mechanization, specialization, and intelligent direction. Based on the predecessor research, this study proposes an artificial neural network model for indoor decoration intelligence calculation and automation design. Based on scales, walls, doors, windows, and other specific components, digital image processing technology implements automatic identification of the apartment graph and completes the preprocessing of the floor plan map. Combined with the indoor decoration data set, the automated design model based on an artificial neural network is established, and the network structure and training process of the model are analyzed. Finally, the bedroom and the living room were experimentally designed. The results showed that as the number of training increased to 30 times, the MAE and MSE assessment indicators gradually decreased, and the error of the model was very small and gradually stabilized. This shows that artificial neural network automation design is better; second, artificial neural network algorithms can generate multiple layout schemes within 1 minute. The design layout is efficient and the plan is reasonable. It meets all requests such as circulation, openness, lighting, and functionality, saving a lot of human and time and providing users with more choices.

## 1. Introduction

As one of the most potential industries, the indoor decoration industry is in the stage of rapid development. Between 2012 and 2017, the overall market size of the interior industry has maintained rapid growth, from 1.5 trillion yuan in 2012 to more than 2 trillion yuan, and the market size of the entire interior decoration industry is expected to reach 2,880.8 billion yuan in 2022. Traditionally, indoor decoration largely relies on the proficiency and technical skills of the staff, often takes a long time, offers users a limited number of options, and cannot meet diverse needs [1]. With people's demand for a good life and living space, traditional indoor decoration cannot meet social needs, and the indoor decoration industry has gradually changed toward mechanization, specialization, and intelligent direction. Using computer technology to implement indoor decoration intelligence calculations and automation will reduce a large amount of human material, providing more personal services for more users.

The article "Artificial Neural Network Model for Indoor Decoration Intelligence Calculation and Automation Design" was published in 2022. Journal: Comput Intell Neurosci.

Hinton proposed a deep neural network model in 2006 that realized the reduction method of data, and the research into neural networks has continued since then [2]. In recent years, deep structural networks have achieved excellent performance in various field applications and have shown the most rapid development in the field of artificial intelligence [3]. Many traditional industries have begun to use artificial intelligence technology for business innovation, so the application of the indoor decoration industry and neural networks will appear with the development of the times. However, there are still many difficult problems. The existing firming graphical identification algorithm is low, the recognition accuracy is low, and the market demand is not met [4]; and the indoor decorative count needs to meet the functionality, aesthetic, comfort, etc. in ergonomics. An automatic layout design algorithm cannot deal with all kinds of complex problems flexibly and cannot realize an intelligent layout.

In summary, this study proposes an artificial neural network model for interior decoration intelligence calculation and automation design. It analyzes the characteristics of the indoor decoration, using artificial neural networks, intelligently calculates the data, and combines the indoor decoration data set to establish an automated design model based on the artificial neural network. This model has broken the interior decoration region restriction, reduces the dependence of people on home improvement, improves the production efficiency of indoor decoration, and can be standardized and transparent. Therefore, the application of artificial neural networks in indoor decoration has high business value and even social value.

## 2. Related Discussion

The interior decoration design is intended to create a spatial structure that meets functional needs. Using artistic methods, by selecting suitable materials, furniture accessories that meet the needs, and suitable decorative styles, the cold architectural space is transformed into a warm space to meet people's comfort requirements for living and working environments [5]. Regarding interior decoration design, some researchers at home and abroad have tried a large number of effective methods and achieved certain results. The early interior decoration design focused on the induction and summary of the home decoration design field by excellent designers, formulated various design rules to realize the decoration design layout, and used CAD (computer-aided design) and 3DMAX and other software to present [6]. Most of the designers are based on the existing mainstream design rules. For example, based on more than 40 years of design experience, Liu and Huilin have compiled the rules of residential design in the book “An Analysis of Residential Design” [7].

The article "Artificial Neural Network Model for Indoor Decoration Intelligence Calculation and Automation Design" was published in 2022. Journal: Comput Intell Neurosci.

In 2015, with the rise of “Internet+,” the residential design model in the Internet era is used to transform the interior decoration design. BIM (Building Information Modeling) has introduced the field of home improvement design [8]. BIM solves the information interaction of traditional design software. BIM technology has a powerful visualization function that can convert the design solution from an abstract two-dimensional drawing to a three-dimensional model and can overcome a variety of modifications [9]. But BIM is designed for indoor decoration, still relying on the designer's experience, and there is also a layout method of BIM. This method is relatively simple, the accuracy is general, and the generalization is poor, susceptible to the room structure. With the external changes such as the room structure, the application scenarios are also changed, resulting in very limited limitations and is limited to complex data. Especially the results of indoor decoration design are affected by designers according to a specific priori knowledge. Therefore, it is impossible to meet the current demand of a large number of fast indoor decoration. Although there are many related fields to explore in the indoor decoration design, it is not enough; there are many problems in the field of indoor decoration that need to be resolved. For example, how to make the interior layout design faster and how to generate various styles of design are worthy of in-depth study and exploration [10]. Therefore, the indoor layout design is done through the computer, making the designer's creations and the ordinary people's lives more meaningful.

In the early stage of interior decoration, there were semi-automatic algorithms. In order to realize full automation, automatic layout algorithm based on rules and scene library was proposed. When the size of the house and the size of the furniture change, it is necessary to modify the rule parameter values manually, and the complex relationship between multiple furniture cannot be defined and processed. The layout of a single furniture may be reasonable, but the overall layout is unreasonable. In order to improve the above shortcomings, algorithms based on intelligence are proposed, and stochastic optimization algorithm and neural network algorithm are the mainstream research direction. A model which can automatically estimate the attitude information of corresponding depth data can be obtained through neural network method training. The model trained by neural network has more objective results than artificial features or algorithms.

The article "Artificial Neural Network Model for Indoor Decoration Intelligence Calculation and Automation Design" was published in 2022. Journal: Comput Intell Neurosci.

In the last century, people have begun to have a certain degree of research on neural networks, and the mechanism of simulate brain cognition is solved. Neural networks have good characteristic learning capabilities, but people know very little about traditional multilayer neural networks, so they cannot solve the problem of conventional multilayer neural networks that cannot converge. As a result, the model may fail to achieve local optimal solutions, so the traditional multilayer neural network cannot be widely applied[11]. With the algorithm of artificial intelligence, Saraei, N., Gupta, and A. J. put forward the pattern of layered training. This can solve the problem of the network being unable to converge to a certain extent [12]. The neural network has now achieved successful applications in image analysis, video categories, natural language processing, and speech recognition [13].

Under the wave of artificial intelligence, the combination of indoor decoration industry and neural network will appear with the development of the times. The artificial intelligence of home decoration soft decoration layout design can assist designers not only to complete a high standard, efficient design scheme and reduce repetitive design steps, but also to reduce the cost of enterprises. As a result, researchers are better able to understand and handle interior decoration design data, enabling them to learn relationships in each data within the interior decoration design. In this context, this study proposes an artificial neural network model for interior decoration intelligence calculation and automation design.

## 3. Construction of Artificial Neural Network Model

The indoor decoration intelligence calculation and automation design is divided into two aspects: one is automatic identification of the apartment graphical identification, that is, automatically identifies all components such as walls, doors, windows, etc., and three-dimensional modeling. The second is the intelligent computing and automation design of the design layout, that is, according to the room function attribute, contour structure, and to-lay furniture, the design layout in the room is automatically completed.

### 3.1. Automatic Identification of a Graph

In the indoor decoration design, the designer needs to prepare the two-dimensional set of graphs, which is based on the information of the apartment pattern, and generates a visual three-dimensional model [14]. This study uses digital image techniques in artificial neural networks to present the automatic identification algorithm of the apartment graph, complete the stage of maltreatment during the layout of the decoration design layout, and automate the three-dimensional modeling.

The article "Artificial Neural Network Model for Indoor Decoration Intelligence Calculation and Automation Design" was published in 2022. Journal: Comput Intell Neurosci.

#### 3.1.1. Frame Diagram Recognition Component

The so-called fellow diagram is automatically identified, and it is to automatically identify the information of the outbound set by the computer. A complete set of figures include walls, doors, and windows; spatial function information; and spatial size information. [15]. These elements have a very important role in three-dimensional reconstruction and subsequent home improvement design, so this summary is to identify these important components (Figure 1).

The components to be identified in the floor plan include scale information and other annotation components, which are used to restore the real size of the space. It also includes contour information such as the position and thickness of structural components such as load-bearing walls and non-load-bearing walls, which are used to build the framework of the 3D model. It also includes functional components such as doors and windows, which makes the effect in the subsequent home improvement design process more reasonable, practical, and beautiful. After completing the identification of the floor plan, you can connect with the 3D modeling platform to generate a visual 3D model for the designer to carry out the next step of interior design layout work.

#### 3.1.2. Frame Diagram Identification Process

This section describes the automatic identification of the individual components of the apartment pattern in accordance with the proportional scale, wall detection, the order of the door, and window recognition.

*(1) Identification of Scale.* Scale, which is the most essential part of plan, determines the scaling of the entire space; the scale identifier include the positioning of the scale endpoint and the identification of the above digits. Finally, the scales can be obtained by the ratio of the identified numbers and pixel lengths [16].

As shown in Figure 2, this study first uses graphics to propose a scale, then divides the above digital image, then identifies the image by a mature open source OCR tool, and finally restores the actual ratio of the entire image. The specific process is, first, after the original image is completed and barbarized; it utilizes morphological operation, extracts all horizontal lines in the image, and the scale to be further identified is the top horizontal line. Then, the top one horizontal line is scanned, the starting point and end coordinates of the scale are obtained, and finally the abscissa to obtain the pixel length is calculated. Next, the intermediate region above the horizontal line is taken, and the rectangular area is identified by the existing digital recognition technique to obtain a scale value. Finally, the ratio of the pixel length and the scale value is used as the zoom ratio of the apartment.

*(2) Wall Detection*. The wall is the most obvious and most basic component in the apartment diagram, which determines the outline structure of the entire space. It has two natures of load-bearing walls and non-loaded walls, and its nature determines whether it can be disassembled during subsequent home improvement. And in the apartment diagram, their difference is whether they are filled by pixels, that is, solid or hollow [17].

The article "Artificial Neural Network Model for Indoor Decoration Intelligence Calculation and Automation Design" was published in 2022. Journal: Comput Intell Neurosci.

For the detection of load-bearing walls and non-supporting walls, the recognition process is as follows:

① Enter the two-value image of the narcotization process;
② Find all connected areas using the Measure module of the Ski mage function library in Python;
③ Find out the external rectangle for each communication area;
④ For all external rectangles, if the area of the rectangle is smaller than the set threshold, the contour of the communication area greater than the set threshold is discarded as the endpoint of the load-bearing wall.

*(3) Identification of Doors and Windows*. The identification of the door has an important role in the three-dimensional rectification of the apartment diagram. It cannot be blocked by furniture during the subsequent decoration design layout. It is an important factor in considering room functionality and practicality during the design [18]. Based on common sense and observation of the floor plan, it can be found that the door and the wall have a relative relationship, that is, the door exists in the wall. In the previous section, we have accurately identified all the walls, so there is no need to identify the doors on the entire image, locate all the candidate areas of the doors through the walls, and then identify the doors on the candidate areas.

A door model graph can show that the door is divided into two kinds: one is a single-opening door and the other is a double-opening door. In the house type drawing, two adjacent and symmetrical single doors form a double door. For the detection of all single doors, if the meeting depends on the same wall, two pairs of inspections shall be conducted: parallel to the wall in the same direction and perpendicular to the wall in the opposite direction. If the distance between them is less than the set threshold, the pair of single doors is determined as double doors and removed from the single door group.

The recognition of windows also plays an important role in the three-dimensional reconstruction of the floor plan. Lighting conditions are an important factor to consider in the subsequent home improvement design process [19]. Similar to doors, windows also depend on and exist in walls. Windows are divided into two types, namely, ordinary windows and bay windows, both of which have a unified drawing mode. A common window consists of two juxtaposed rectangles (Figure 3), while a bay window consists of three rectangles that share a long side. So, the window recognition process is

① The Open's Minaret function is used to get all the internal rectangular rectangles in the unit drawings
② When the vertical distance between the long edges is less than the set threshold, it is judged as a public window.
③ When two or more internal rectangles share a long side, the distance between the short sides of the inner rectangle is smaller than the set threshold, which is judged as a slave

The article "Artificial Neural Network Model for Indoor Decoration Intelligence Calculation and Automation Design" was published in 2022. Journal: Comput Intell Neurosci.

### 3.2. Design Layout Intelligence Computing and Automation

In response to the lowest response speed of the indoor decoration, the advantages of artificial neural networks are used in the advantages of artificial neural network, and the model is used to train the model based on the existing layout design scheme data set. The model can automatically generate information such as the coordinate point of the decoration design layout, while the upper limit of the model and the prediction accuracy of the design layout are affected by the data sample. Therefore, the data are selected and handled before the training model.

#### 3.2.1. Data Set

The nature of the neural network is from *N*-dimensional spaces to *M*-directional nonlinear mapping, and the neural network model passes the training process, and the layout design can be properly predicted. Features are important factors affecting the design accuracy of indoor layout [20]. In order to better extract and process features from the data used, the feature project is used to process the data set. The pres-treatment is mainly analyzed for the screening and design of the design and screening input variables, and the bedroom feature data are shown in Table 1.

#### 3.2.2. Data Feature Processing

In the field of artificial neural network, the characterization determines the upper limit of the model, so feature extraction becomes an indispensable link in the design of decoration layout [21]. Although the decoration layout is designed to have many features, not all features are necessary for indoor decoration design applications, and below for the characteristics of indoor decoration design [22].

(1) Americanization of qualitative feature: For design style features and room structural features, transformation into numbers represents design style and room structural features and facilitates the input of variables. The following are the conversion formulas of style characteristics, the conversion formula of bedroom structure, and the conversion formula of living room structure.
  (1) $$\begin{array}{c} a=\left\{\begin{array}{c} 0,\text{ European style,}\\ 1,\text{ Chinese style,}\\ 2,\text{ Simple style,} \end{array}\right)\\ a=\left\{\begin{array}{c} 0,\text{ Vertical hall type,}\\ 1,\text{ Horizontal hall type,} \end{array}\right)\\ a=\left\{\begin{array}{c} 0,\text{ mouth font,}\\ 1,\text{ L shape.} \end{array}\right) \end{array}$$
where *a* represents the parameter that decorates the structure of style, sitting room, and bedroom structure.
(2) Combination characteristics: Processing of raw characteristics and generating new feature variables. According to the location of the bedroom door and the position of the bed, the relative distance of the door and the bed is created, the two new features of the door direction and the heading of the bed are also created.
  (2) $$\begin{array}{c} a=\sqrt{{\left(a_{1}-a_{2}\right)}^{2}+{\left(b_{1}-b_{2}\right)}^{2}}, \end{array}$$
where *a*_1_ and *b*_1_ are the points of the door, *a*_2_ and *b*_2_ are the points of the bed.
  (3) $$\begin{array}{c} a=a_{1}\times a_{2}+b_{1}\times b_{2}, \end{array}$$
where *a*_1_ and *b*_1_ are the direction vectors of the door, and *a*_2_ and *b*_2_ are the head vectors.
People have a sufficient demand for the bedroom light, and the location of the usual bed is often close to the window. At the same time, the designer in the bedroom design is in order to facilitate the user and adaptation of the user's usage habits, usually put the wardrobe layout directly on the bed side; the position of the bed directly affects the layout position of the wardrobe, thereby creating a new feature of the relative distance of the bed and wardrobe. Based on the above analysis, the following formula is obtained:
  (4) $$\begin{array}{c} a=\sqrt{{\left(a_{1}-a_{2}\right)}^{2}+{\left(b_{1}-b_{2}\right)}^{2}}, \end{array}$$
where *a*_1_ and *b*_1_ are window coordinates or bed coordinates, *a*_2_ and *b*_2_ are bed coordinates or wardrobe point coordinates.
In the bedroom design, designers tend to choose the size of the decoration design according to the room area. Then the size of the room area and the decoration design is directly related, and creating a room area is compared to the new features of the width of the bed, which is expressed as
  (5) $$\begin{array}{c} a=\left(\frac{\text{area}}{\text{width}}\right)\times 100\%, \end{array}$$
where area is the room area, width is the width of the bed, and the unit is rice.
After the original feature is treated, the new feature data of the bedroom is shown in Table 2.
(3) Standardization: data set samples are different, the room structure coordinate in the design does not agree, causing the difference between each sample, thus turning the sample coordinates to the same coordinate.
(4) Normalization of data: since the length of the storage unit of each sample is not used, the length information of the sample in the data set is first in units of centimeters, and the area is in square meters. Since variables for different design layout samples typically have different dimension and dimension units, this situation directly affects data analysis and input parameters of neural networks. By standardizing the data, we eliminate the dimension influences between different indoor layout design sample parameters, and therefore, we process the design sample data for the decoration design layout using *Z*-score standardization, which is expressed as
  (6) $$\begin{array}{c} a=\left(\frac{\left(a-\bar{a}\right)}{\beta }\right). \end{array}$$

The *a* is the mean of data in the formula, and *β* is the standard deviation of data.

The article "Artificial Neural Network Model for Indoor Decoration Intelligence Calculation and Automation Design" was published in 2022. Journal: Comput Intell Neurosci.

#### 3.2.3. Model Structure

Since the layout is designed with multiple point coordinate information, the artificial neural network is applied to the generation of indoor decoration design layout, and the output of the neuron of each output represents a dimension of a point coordinate. The network structure is shown in Figure 4.

As shown in Figure 4, the input layer passes through different hidden layer combined structures, and the ability to describe different outputs is fully utilized, and the prediction capability of the entire network is improved. The implicit layer is mainly for constant learning characteristics, and the number of implicit layers of the network affects the results of the forecast. If the number of layers are not better than the traditional neural network, excessive number of layers will lead to a decline in learning efficiency. The hidden layers of this study select three layers and have multiple separate network structural sections, each connected to an output layer node, respectively. The number of input layer neurons of the model is *X*, and the number of output layer neurons is *Y*. This structure has given the ability to describe the description of different characteristics and improve the generalization of the model, thereby improving the performance of the network.

#### 3.2.4. Model Training

(1) The *i* sample is used as an input variable *v* of the model, and the implicit layer corresponding to the sample can be calculated as follows:
  (7) $$\begin{array}{c} y_{oh}=\sum_{o=1}^{n}w_{hk}v_{i}+b_{h}. \end{array}$$
(2) The error of the model is calculated as follows:
  (8) $$\begin{array}{c} F=\frac{1}{2}\sum_{o=1}^{n}{\left(v_{i}-v_{\text{oh}}\right)}^{2}\\ =\frac{1}{2}\sum_{o=1}^{n}\left(w_{hk}v-\text{b}\right)+b_{h}. \end{array}$$
(3) The bias number of F is calculated as
  (9) $$\begin{array}{c} \alpha \frac{y_{oh}}{w_{oh}}=\frac{\alpha \left(\sum_{o=1}^{n}w_{hk}v_{i}+b_{h}\right)}{\alpha w_{oh}}. \end{array}$$
(4) According to the learning rate and according to the method of decrease the gradient, the weight between each layer in the model and the bias between the layers and the layers are decorated, which is represented as follows:
  (10) $$\begin{array}{c} \Delta w_{oh}=\pm \lambda \left(\frac{\alpha F}{\alpha w_{oh}}\right)\Rightarrow w_{oh}^{i+1}, \end{array}$$
where *λ* represents the learning rate.
(5) The weight and threshold of reactive artificial neural network model are used after updating by the learning rate, and the next error calculation is performed. If the error result meets the threshold of the network or the number of learning times of network settings, the network stops training, otherwise the model will continue to train until the requirements of network settings are met.

The article "Artificial Neural Network Model for Indoor Decoration Intelligence Calculation and Automation Design" was published in 2022. Journal: Comput Intell Neurosci.

## 4. Model Design Layout Experiment Design

### 4.1. Experimental Design

This experiment uses the interior design layout data set after the characteristic engineering. According to the indoor design characteristics and room structure, the experiment divides the data set into two major categories, namely the bedroom data set and the living room data set. Data sets of each part are trained, and the design layout model based on artificial neural design layout model is experimentally analyzed by the experimental results displayed by the index. The experiment configuration is shown in Table 3.

Software environment: Cuda, Caffe, Python, Ubuntu 14.04 LTS.

### 4.2. Evaluation Indicator

This study introduces two different evaluation metrics to measure the performance of artificial neural network model in interior decoration layout design prediction. Two evaluation criteria are: mean squared error (MSE) and mean absolute error (MAE). MSE and MAE evaluate the model from the perspective of the prediction error of the interior decoration design layout, reflect the error of the entire model prediction, and can illustrate the level of the model's prediction ability. The evaluation indicator is shown in Table 4.

The process of furniture layout requires ergonomics, aesthetics, functionality, and other aspects. Therefore, this study also adds eight evaluation indexes of average time consumption, circulation, openness, room vacancy rate, day lighting, functionality, minimum correction steps, and minimum correction time.

The article "Artificial Neural Network Model for Indoor Decoration Intelligence Calculation and Automation Design" was published in 2022. Journal: Comput Intell Neurosci.

## 5. Results and Analysis

### 5.1. Design Index Evaluation Analysis

In the whole process of interior decoration, the living room and bedroom occupy more than 80% of the total area, and the living room and bedroom are the place where people spend the longest time. Therefore, their importance in the decoration process is obvious. According to the data set, the experimental results are divided into bedrooms and living room. By MSE, MAE evaluates the prediction of indoor layout design model based on the artificial neural network. The bedroom data set is used as training data, introduced into the MAE and MSE evaluation indicators.  Table 5 shows the results of predictive assessment index of the design layout model based on the artificial neural network.

As can be seen from Table 5, the MAE and MSE values of the *X* coordinate of the bed are large. The model has a certain error on the prediction of the bed in the position of the *X*-axis in the room, the evaluation index of other parameters is small, and the model has a certain error. But overall, the prediction effect of the decoration design layout of the bedroom is better.

As can be seen from Figure 5, there is a significant convergence after the network iteration, and the MAE and MSE evaluation indicators gradually decrease as the number of training times is 30 times, and the error of the model is very small and tends to stabilize.

The vertical hall living room data set is used as training data, and MAE and MSE evaluation indicators are introduced.  Table 6 shows the layout prediction evaluation index of the decoration design layout model based on the artificial neural network.

As can be seen from Table 6, the MAE and MSE values of the sofa combination *X* coordinate are large. The model is better to the sofa combination, and there is still a large prediction error of the sofa combination in the room coordinate system *X* coordinates.

As can be seen from Figure 6, MAE has a significant convergence about 3 times in the network, and MSE tends to be stable on the network iteration, and the number of iterations increases the MAE and MSE evaluation indicators.

Through the experiment of the bedroom and living room automation layout, the experimental results show that the decoration design layout model based on the artificial neural network has a good effect on the prediction of the indoor design point.

### 5.2. Design Plan Comparative Analysis

The experimental data used in this study are 500 sets of good layout schemes provided by several professional interior design companies, and the file format is JSON. First of all, the 500 sets of layout plan are in accordance with the rules introduced before the collision out of the boundary for artificial disruption, including disruption of very individual and disruption of multiple furniture, furniture small range or large range out of the boundary, and slight collision between furniture or serious collision. Each scheme was randomly shuffled for 10 times of varying degrees, and a total of 5000 schemes were generated to be scored. Then let a number of professional home decoration designers evaluate the scheme and give a score, and the average is taken of all points as the score of the furniture layout scheme.

The article "Artificial Neural Network Model for Indoor Decoration Intelligence Calculation and Automation Design" was published in 2022. Journal: Comput Intell Neurosci.

This experiment demonstrates the two-dimensional renderings of the bedroom layout based on the strategic algorithm and artificial neural network algorithm, where the dashed portion is the main area divided into the pres-processing step. The layout effect is shown in Figure 7.

Compare the average time, cycle, openness, room vacancy rate, lighting, function, minimum correction step, and minimum correction time of the two algorithms, and the conclusion is shown in Figure 8.

As can be seen from Figure 8, the automatic layout algorithm based on the artificial neural network model is obviously superior to the algorithm based on strategy gradient in terms of real-time performance and can also meet the requirements of fluidity, openness, vacancy rate, day lighting, functionality, etc.

The purpose of this algorithm is to generate layout scheme automatically and save designers a lot of layout and adjustment time. After the automatic layout, the designer can make small adjustments manually. The minimum number of corrected steps refers to the minimum number of steps that the designer manually adjusts to meet a requirement based on an automatically generated layout scheme. Minimum correction time refers to the minimum adjustment time that the designer manually adjusts the layout scheme based on automatic generation.

This experiment demonstrates the two-dimensional renderings of the living room layout based on the strategic algorithm and artificial neural network algorithm, where the dashed portion is the main body area divided into the pres-process step. The layout is shown in Figure 9.

Extending the rationality index of the bedroom, the layout design of the living room is analyzed and the layout results are compared with the algorithm based on the strategy gradient. The comparison of each evaluation index is shown in Figure 10.

As can be seen from Figure 10, the artificial neural network algorithm is equipped to generate multiple sets of design within 1 minute. The design is reasonable, which can meet the requirements of circulation, openness, lighting, and functionality. In the layout design of the living room, the user's visual balance is met. After the layout plan, the professional designer only needs to fine-tune, which can complete the layout design of the room, saving a lot of manpower and time, and can provide users with more *s* Choice.

The article "Artificial Neural Network Model for Indoor Decoration Intelligence Calculation and Automation Design" was published in 2022. Journal: Comput Intell Neurosci.

This section has conducted experiments and tests for the rooms of different profile structures and different functional properties, and the design schedule was evaluated using multiple evaluation indexes. The algorithm does not need to model the intelligent body and the environment feedback model, saves time, improves efficiency, and can generate a reasonable design. The experimental results prove the effectiveness and efficacy of the algorithm.

## 6. Conclusion

Under the current labor intelligence, industrial structure upgrade in the indoor decoration design has brought innovation points. Based on the current technology trend, this article studies the artificial intelligence in the indoor decoration layout design area and explores the indoor decoration intelligence calculation and layout design through artificial neural network models, helping designer creation and ordinary people to decorate design. Through experiments, the effectiveness and practicality of the artificial neural network models in the indoor decoration layout design, saving a large number of human and time, can provide users with more choices. At present, the target users of this mode in the field of intelligent decoration design are middle and low-end users, while high-end users are still served one to one by senior designers. In the future, we hope to extend this model to advanced users and improve the novelty and uniqueness of layout design [22].

## Figures and Tables

**Figure 1:** Frame diagram recognition component.

**Figure 2:** Scale identification extraction map.

**Figure 3:** Identification diagram of doors and windows.

**Figure 4:** Network structure diagram.

**Figure 5:** (a) MAE and (b) MSE evaluation indicator of the bedroom.

**Figure 6:** (a) MAE and (b) MSE evaluation indicators of the living room.

**Figure 7:** Bedroom layout renderings.

**Figure 8:** Bedroom layout plan comparison.

**Figure 9:** Living room layout renderings.

**Figure 10:** Living room layout plan comparison.

**Table 1:** Bedroom feature data sheet.

Basic parameters	Wall structure	Door position	Wardrobe spot
Parameter definition	Room wall spot	Door opening point, rotation point	Define the direction vector according to the plan coordinate system
Expression form (cm)	(*a*, *b*)	(*a*, *b*)	(*a*, *b*)
Basic parameters	Door opening direction	Window point	Wardrobe orientation
Parameter definition	Defined according to the floor plan	The structural center point of the window	Define the direction vector according to the plan coordinate system
Expression form (cm)	(0, 1); (0, −1); (1, 0); (−1, 0)	(*a*, *b*)	(0, 1); (0, −1); (1, 0); (−1, 0)
Basic parameters	Bed position	Bed orientation	Room size
Parameter definition	Take the upper left point of the bed as the reference point of the bed	Define the direction vector according to the plan coordinate system	Take the total area of the room
Expression form (cm)	(*a*, *b*)	(0, 1); (0, −1); (1, 0); (−1, 0)	*a*
Basic parameters	Design style	Room structure	
Parameter definition	Simple style, European style, and Chinese style	Mouth type, L type	
Expression form (cm)	0, 1, 2	0, 1	

The article "Artificial Neural Network Model for Indoor Decoration Intelligence Calculation and Automation Design" was published in 2022. Journal: Comput Intell Neurosci.

**Table 2:** New feature data sheet.

Basic parameters	The relative distance between the door	Door orientation and bed orientation
Expression form (cm)	*a*	(*a*, *b*)
Basic parameters	Bed window relative distance direction	Relative distance between bed and wardrobe
Expression form (cm)	*a*	*a*
Basic parameters	Room size and bed size	Wardrobe orientation and room structure
Expression form (cm)	*a*	(*a*, *b*)

**Table 3:** Experimental configuration table.

Operating platform	Windows
CPU	Intel(R) XEON(R) CPU I7- 6800K @ 2.00 GHz (28 cores, 56 threads)
RAM	128 GB
GPU	NVIDIA GEFORCE GTX1080Ti
Survive	12 GB
Hard disk	3.1 TB SSD

**Table 4:** Evaluation indicator table.

Predicting category	Indicator content
MSE	Identify the sum of squared distances between the experimental predicted value and the true value average
MAE	Identify the absolute difference between the experimentally predicted value and the true value sum of values.

**Table 5:** Predictive evaluation index.

Parameter	bed_point_a	bed_point_b	bed_vex_a	bed_vex_b	wardrobe_point_a	wardrobe_point_b	wardrobe_vex_a	wardrobe_vex_b
MSE	7.063625	0.938556	0.625576	0.138538	1.784406	0.449938	0.515152	0.153733
MAE	68.723175	0.234486	0.044431	0.032170	0.488192	0.034345	0.026530	0.036326

**Table 6:** MAE and MSE evaluation indicators of the living room.

Parameter	sofa_point_a	sofa_point_b	sofa_vex_a	sofa_vex_b	TV bench__point_a	TV bench_point_b	TV bench_ vex_a	TV bench_ vex_b
MSE	6.896639	1.059642	0.427846	0.072872	0.355298	1.138977	0.152303	0.095198
MAE	67.684661	1.706067	0.424330	0.095851	0.205701	2.104715	0.039421	0.018186

## Data Availability

The data used to support the findings of this study are available from the corresponding author upon request.
